# LncRNA miR503HG interacts with miR-31-5p through multiple ways to regulate cancer cell invasion and migration in ovarian cancer

**DOI:** 10.1186/s13048-019-0599-9

**Published:** 2020-01-06

**Authors:** Ding Zhu, Xueshuang Huang, Fang Liang, Lijing Zhao

**Affiliations:** 1 Department of Gynecology, Hunan Provincial People’s Hospital, Changsha City, Hunan Province 410005 People’s Republic of China; 2 Biomedical Research Center, Hunan University of Medicine, No.492 Jinxi South Road, Huaihua City, Hunan Province 418000 People’s Republic of China

**Keywords:** Ovarian cancer, miR503HG, miR-31-5p, Prognosis

## Abstract

The role of lncRNA miR503HG has been investigated in several types of cancer, but its functions in ovarian cancer (OC) is unclear. Analysis of TCGA dataset revealed a 50-fold lower expression level of miR503HG in OC tissues than that in non-tumor tissues, indicating the involvement of miR503HG in OC. Results in this study showed that miR503HG was downregulated in OC and predicted poor survival. Expression of miR503HG negatively correlated with the expression of miR-31-5p across OC and non-tumor tissues. RNA-RNA interaction analysis revealed that miR503HG can interact with miR-31-5p. Dual-luciferase assay showed that miR-31-5p and miR503HG may directly interact with each other. Methylation specific PCR (MSP) showed that overexpression of miR503HG led to increased methylation level of miR-31-5p gene. Transwell assay showed that overexpression of miR-31-5p resulted in increased invasion and migration rates of OC cells. Overexpression of MiR503HG played an opposite role and attenuated the effects of overexpressing miR-31-5p. Therefore, miR503HG may promote the methylation of miR-31-5p and serve as its sponge to inhibit OC cell invasion and migration.

## Introduction

Ovarian cancer (OC) is one of the most common types of female cancers and a leading cause of cancer-related deaths [1]. According to the latest GLOBOCAN statistics, OC caused 184,799 deaths (1.9% of all cancer deaths), and affected 295,414 new cases (1.6% of all new cancer deaths) [2]. Even with the advanced treatments of OC, survival of patients is generally poor, mainly because most patients were diagnosed at advanced stages with metastatic tumors [3]. Aging and obesity have been proven to be the major risk factors for OC [4, 5]. However, molecular pathogenesis of OC remains unknown.

The emergence of targeted therapies provided novel insights into the treatment of OC [6, 7]. However, the lack of effective and safe targets limited the clinical applications. Besides protein coding genes, non-coding RNAs (ncRNAs) are also critical players in cancer biology and they mainly function through the regulation of cancer-related genes [8, 9]. Therefore, regulation of cancer-related ncRNAs may be beneficial for cancer control and treatment [10]. Long (> 200 nt) non-coding RNA (lncRNA) miR503HG has been characterized as a tumor suppressor in hepatocellular carcinoma and large-cell lymphoma [11, 12]. Analysis of the cancer genome atlas (TCGA) database identified that miR503HG was significantly downregulated in OC compared to non-tumor tissues. In addition, miR503HG was predicted to interact with miR-31-5p, which has been reported to play oncogenic roles in various types of cancer [13]. However, the involvement of miR503HG in OC and its potential interaction with miR-31-5p remain unknown. This study was carried out to investigate the involvement of miR503HG and miR-31-5p in OC.

## Materials and methods

### OC patients

The Hunan University of Medicine admitted 109 OC patients (high-grade serous carcinoma) from January 2011 to July 2014, and 61 patients (all Chinese females, 36–67 years old, with the mean age of 53.1 ± 6.0 years old) were selected in this study. Inclusion criteria: 1) newly diagnosed OC patients; 2) no initiated therapies before this study. Exclusion criteria: 1) recurrent cases; 2) other severe clinical disorders were observed; 3) therapies were initiated before the study. Informed consent was obtained from each patient and the study was approved by the Ethics Committee of Hunan University of Medicine. All patients were informed of experiments involved in this project and written form informed consent was provided by all of them.

### Biopsies and treatment

Ovarian biopsy was performed on all 61 OC patients under the guidance of MRI before any therapies. OC biopsy was collected to diagnose OC by histopathological examinations. Non-tumor tissues adjacent (within 3 cm around tumors) were also collected during biopsy. All biopsies were confirmed by histopathological exams. The 61 patients were staged according to the AJCC criteria. There were 12, 16, 16 and 17 cases at clinical I, II, III and IV, respectively. According to clinical stages, the patients were treated with surgical resection, radiation therapy, chemotherapy or their combinations.

### Follow-up

From the day of admission, all 61 OC patients were followed up for 5 years. In most cases patients were visited by phone calls. In some cases, outpatient visits were also included. The patients lost contacts or died of other causes were excluded in the survival analysis.

### OC cell lines and transfections

Two human OC cell lines, UWB1.289 (ATCC, USA) and A2780 (Sigma-Aldrich), were used as the cell model of OC. Cells of both cell lines were cultivated in a mixture of 10% FBS and 90% RPMI-1640 medium. Cells were cultured at 37 °C with 5% CO_2_ and 95% humidity. Cells were harvested at 70–80% confluence to perform transfections. The miR503HG expressing vector was constructed using pcDNA3.1 vector (RIBOBIO, Guangzhou, China). Negative control (NC) miRNA and miR-31-5p mimic were obtained from Sigma-Aldrich. UWB1.289 and A2780 cells (2 × 10^6^) were transfected with 10 nM vector (NC group was the empty vector) or 50 nM miRNA (NC group was the NC miRNA) using lipofectamine 2000 (RIBOBIO). Three biological replicates were set for each transfection. Untransfected cells were used as Control (C) cells in all transfections. Cells harvested at 24 h post-transfection were used in all subsequent experiments.

### Dual-luciferase assay

The interactions between miR503HG and miR-31-5p were investigated by dual-luciferase assay. In this assay, transfections were performed through the same way as aforementioned except that psiCHECK-1 vector (Promega), instead of pcDNA3.1 was used. Cells were transfected with either miR503HG + miR-31-5p or miR503HG + NC miRNA. Three biological replicates were set for each transfection. Renilla luminescence was normalized by firefly luminescence.

### RNAs extractions and qPCR

All biopsies from 61 OC patients were ground in liquid nitrogen. UWB1.289 and A2780 cells were harvested at 24 h post-transfection. RNAzol (Sigma-Aldrich, USA) was used to extract total RNAs from 0.03 g biopsy or 2 × 10^5^ cells. To harvest miRNAs, RNA samples were precipitated using 85% ethanol. With poly (T) as primer, cDNA was synthesized through reverse transcriptions (RTs) using PrimeScript RT Reagent Kit (Takara, Japan) with 1 μg RNA as template. qPCR reactions were performed using the SYBR Green Master Mix (Bio-Rad). The expression level of miR503HG was normalized to endogenous control 18S rRNA. Expression levels of mature miR-31-5p were evaluated by addition of poly (A), RTs and qPCR assays. All steps were completed using All-in-One™ miRNA qRT-PCR Detection Kit (GeneCopoeia, Guangzhou, China). The expression level of miR-31-5p was normalized to U6. All PCR reactions were repeated 3 times and the 2^-ΔΔCT^ method was used for all data normalizations.

### Methylation-specific PCR (MSP)

Genomic DNA Extraction Kit (ab156900, Abcam) was used to extract genomic DNAs from both UWB1.289 and A2780 cells. Methylation-Gold™ kit (ZYMO) was used for bisulfite conversion. MSP reactions were performed using Taq DNA polymerase (NEB).

### Transwell assays

The effects of transfections on the invasion and migration of UWB1.289 and A2780 cells were evaluated by Transwell assays. Cell pellets containing 3 × 10^4^ cells were resuspended in 1 ml non-serum culture medium. Upper Transwell chamber was filled with 0.1 ml cell suspension, and the lower chamber was filled with a mixture of 80% RPMI-1640 medium and 20% FBS. Three chambers replicates were set for each experiment. The Corning Matrigel (200 mg/ml, Corning) was used to coat the membranes at 37 °C for 12 h before use. Cells were cultured for 24 h. The lower surface of membranes was then stained with 0.1% crystal violet (Corning). Cell invasion and migration were observed under a light microscope. The Image J v1.46 software was used to count cells.

### Statistical analysis

Mean values of 3 biological replicates included in each experiment were calculated and used in all data analyses. Correlations were analyzed by linear regression. Differences between two types of biopsies were analyzed by paired t test. ANOVA (one-way) and Tukey test were used to explore differences among multiple groups. To perform survival analysis, the 61 OC patients were divided into the high (*n* = 31) and low (*n* = 30) miR503HG level groups. Survival curves were plotted (K-M plotter) and compared (log-rank test). *p* < 0.05 was statistically significant.

## Results

### Downregulation of miR503HG predicted poor survival of OC patients

Analysis of the TCGA dataset showed that expression level of miR503HG in OC tissues was more than 50 times lower in OC tissues compared to that in non-tumor tissues (1.76 vs. 88.23). To further confirm its downregulation in OC, qPCR was performed to measure the expression levels of miR503HG in both OC and non-tumor biopsies from all 61 OC patients included in this study. The results showed that expression levels of miR503HG were significantly lower in OC than that in non-tumor tissues (Fig. 1a, *p* < 0.05). Comparing to patients in the high miR503HG level group, patients in the low miR503HG level group had significantly lower overall survival rate (Fig. 1b).

**Fig. 1:** Downregulation of miR503HG predicted poor survival of OC patients. qPCR was performed to measure the expression levels of miR503HG in both OC and non-tumor biopsies from the 61 OC patients included in this study. Differences in expression levels between OC and non-tumor biopsies were explored using paired t test (**a**). To perform survival analysis, the 61 OC patients were divided into the high (*n* = 31) and low (*n* = 30) miR503HG level groups. Survival curves were plotted using K-M plotter and compared by log-rank test (**b**). PCR reactions were repeated 3 times and mean values were presented, *p* < 0.05

### MiR503HG may interact with miR-31-5p

The interaction between miR503HG and miR-31-5p was predicted by IntaRNA (http://rna.informatik.uni-freiburg.de/IntaRNA/Input.jsp). It showed that miR503HG could form strong base pairing with miR-31-5p (Fig. 2a). Dual-luciferase assay showed that comparing to cells transfected with miR503HG and NC miRNA (NC), the relative luciferase activity was significantly lower in cells transfected with miR503HG and miR-31-5p (miR-31-5p).

**Fig. 2:** MiR503HG may interact with miR-31-5p. The interaction between miR503HG and miR-31-5p was predicted by IntaRNA (http://rna.informatik.uni-freiburg.de/IntaRNA/Input.jsp). It was observed that miR503HG may form strong base pairing with miR-31-5p (**a**). To confirm the interaction between these two factors, dual-luciferase assay was performed by transfecting miR503HG + miR-31-5p (miR-31-5p) or miR503HG + NC miRNA (NC) into UWB1.289 and A2780 cells (**b**). Experiments were repeated 3 times and mean values were presented. *, *p* < 0.05

### MiR-31-5p was upregulated in OC and inversely correlated with miR503HG

qPCR results showed that expression levels of miR-31-5p were significantly higher in OC tissues than that in non-tumor tissues (Fig. 3a, *p* < 0.05). Correlations between miR-31-5p and miR503HG were analyzed by linear regression and the results revealed that miR-31-5p and miR503HG were significantly and inversely correlated with each other across both OC (Fig. 2b) and non-tumor (Fig. 2c) tissues.

**Fig. 3:** MiR-31-5p was upregulated in OC and inversely correlated with miR503HG. qPCR was performed to measure the expression levels of miR-31-5p in both OC and non-tumor biopsies from the 61 OC patients included in this study. Differences in expression levels between OC and non-tumor biopsies were explored using paired t test. Expression levels of miR-31-5p were significantly higher in OC than in non-tumor tissues (**a**). Correlations between miR-31-5p and miR503HG across both OC (**b**) and non-tumor (**c**) tissues were analyzed by linear regression. PCR reactions were repeated 3 times and mean values were presented, *p* < 0.05

### MiR503HG downregulated miR-31-5p through methylation

To further analyze the relationship between miR-31-5p and miR503HG, UWB1.289 and A2780 cells were transfected with miR-31-5p mimic or miR503HG expression vector. Overexpression of miR-31-5p and miR503HG was confirmed by qPCR. Compared to C and NC groups, expression levels of miR-31-5p and miR503HG were significantly increased at 24 h post-transfection (Fig. 4a, *p* < 0.05). In addition, overexpression of miR503HG resulted in downregulation of miR-31-5p (Fig. 4b, *p* < 0.05). However, overexpression of miR-31-5p did not affect the expression of miR503HG (Fig. 4c, *p* < 0.05). MSP was performed to analyze the effects of overexpressing miR503HG on the methylation of miR-31-5p gene. It showed that overexpression of miR503HG resulted in increased methylation of miR-31-5p gene (Fig. 4d).

**Fig. 4:** MiR503HG downregulated miR-31-5p through methylation. UWB1.289 and A2780 cells were transfected with miR-31-5p mimic or miR503HG expression vector. Overexpression of miR-31-5p and miR503HG was confirmed by qPCR (**a**). The effects of the overexpression of miR503HG on miR-31-5p expression were analyzed by qPCR (**b**). The effects of overexpressing miR-31-5p on miR503HG expression were also evaluated by qPCR (**c**). MSP was performed to analyze the effects of verexpressing miR503HG on the methylation of miR-31-5p gene (**d**). Experiments were repeated 3 times and mean values were presented. *, *p* < 0.05

### MiR503HG suppressed OC cell invasion and migration through miR-31-5p

Transwell assays were performed to analyze the effects of overexpressing miR503HG on cell invasion (Fig. 5a) and migration (Fig. 5b) of UWB1.289 and A2780 cells. Compared to C and NC groups, overexpression of miR-31-5p resulted in increased invasion and migration rates of OC cells. Overexpression of miR503HG played an opposite role and attenuated the effects of overexpressing miR-31-5p (*p* < 0.05).

**Fig. 5:** MiR503HG suppressed OC cell invasion and migration through miR-31-5p. Transwell assays were performed to analyze the effects of overexpressing miR503HG on the invasion (**a**) and migration (**b**) of UWB1.289 and A2780 cells. Experiments were repeated 3 times and mean values were presented. *, *p* < 0.05.

## Discussion

In this study, the functions of miR503HG involved in OC were investigated. Our results showed that miR503HG was significantly downregulated in OC and was closely correlated with poor survival. In addition, miR503HG may attenuate the oncogenic functions of miR-31-5p in OC.

The downregulation of miR503HG has been reported in hepatocellular carcinoma (HCC) and large-cell lymphoma [11, 12]. Analysis of the TCGA public dataset confirmed the downregulation of miR503HG in HCC (0.55 vs. 2,1) and lymphoma (0.62 vs. 4.06) compared to the non-tumor tissues. Downregulation of miR503HG was observed in most types of cancer with fewer exceptions, such as adenoid cystic carcinoma (15.44 vs. 6.69) and glioblastoma (3.39 vs. 0.97). To our surprise, the most significant downregulation of miR503HG was observed in OC (1.76 vs. 88.23), while no previous studies have reported the involvement of this lncRNA in OC. To the best of our knowledge, this is the first study that confirmed the downregulation of miR503HG in Chinese patients with OC. However, the fold change of downregulation of miR503HG in the patients included in this study was only less than 8-fold. This is possibly due to the different populations.

MiR-31-5p has been reported to play oncogenic roles in various types of cancer, such as renal cell carcinoma, colorectal cancer and oral squamous cell carcinoma [13–15]. However, its functions in OC remain unknown. In this study we showed that miR-31-5p was upregulated in OC and promoted cancer cell invasion and migration. Therefore, miR-31-5p is likely an oncogenic lncRNA in OC. We showed that miR-31-5p can bind to miR503HG, while overexpression of miR-31-5p did not affect the expression of miR503HG. Therefore, miR503HG is unlikely a downstream target of miR-31-5p. It was reported that lncRNAs may serve as the sponge of miRNAs [16], which made us to hypothesize that miR503HG might sponge miR-31-5p. However, miRNA sponges usually do not involve the downregulation of miRNAs. Interestingly, overexpression of miR503HG resulted in the downregulation of miR-31-5p. In addition, overexpression of miR503HG also resulted in the increased methylation of miR-31-5p gene. Therefore, miR503HG may attenuate the oncogenic effects of miR-31-5p in OC through two different ways.

It is worth noting that the sample size of this study is relatively small. Also, animal model experiments were not included to further confirm our conclusions. Future studies with bigger sample size and OC animal models are needed to further confirm our conclusions.

In conclusion, miR503HG was downregulated in OC and may suppress OC by increasing the methylation of miR-31-5p gene and sponging mature miR-31-5p.

## Data Availability

The analyzed data sets generated during the study are available from the corresponding author on reasonable request.
